The article "Imaging Signs for Determining Surgery Timing of Acute Intestinal Obstruction" was published in 2022. Journal: Contrast Media Mol Imaging.

# Imaging Signs for Determining Surgery Timing of Acute Intestinal Obstruction

**DOI:** 10.1155/2022/1980371

**Published:** 2022-07-19

**Authors:** Zhenkai Li, Liangliang Shi, Jianhua Zhang, Qiang Sun, Weidi Ming, Zhengming Wang, Hongzhi Sun

**Affiliations:** ^1^Suzhou Medical College of Soochow University, Suzhou, China; ^2^Department of General Surgery, PLA Rocket Force Characteristic Medical Center, Beijing, China; ^3^Department of Hepatobiliary Surgery, PLA Rocket Force Characteristic Medical Center, Beijing, China; ^4^Department of Radiology, PLA Rocket Force Characteristic Medical Center, Beijing, China; ^5^Department of General Surgery, The First Affiliated Hospital of Jinzhou Medical University, Jinzhou, China

## Abstract

We aimed to analyze the computed tomography (CT) imaging signs of bowel wall ischemia in patients with acute intestinal obstruction and construct an imaging prediction model to guide clinical treatment. The CT imaging signs of patients with acute intestinal obstruction diagnosed in our center in recent 6 years were collected for retrospective analysis. The etiology of intestinal obstruction and incidence rate of bowel wall ischemia were recorded, and the specific CT findings of bowel wall ischemia, including mesenteric edema, bowel wall thickening, and fish tooth sign, were analyzed. Among the 302 patients selected, 130 surgically treated patients were eligible for analysis. Bowel wall ischemia in acute intestinal obstruction showed an incidence rate of 14.90%, and the incidence rates of bowel wall ischemia in intra-abdominal hernia, intussusception, incarcerated external abdominal hernia, and volvulus were about 92.30%, 50%, 35.71%, 33.33%, and 12.59%, respectively. The incidence rate of bowel wall ischemia in simple adhesive intestinal obstruction was about 12.59%, and that in malignancy-induced intestinal obstruction was about 6.56%. Univariate analysis revealed 5 factors with statistical significance, including bowel wall thickening, mesenteric edema, bowel wall pneumatosis, ascites, and fish tooth sign. Multivariate logistic regression analysis indicated that fish tooth sign, bowel wall thickening, and mesenteric edema were able to predict bowel wall ischemia, and the corresponding partial regression coefficients were 2.164, 1.129, and 1.173, odds ratios (ORs) were 8.707, 3.093, and 3.232, sensitivity was 0.356, 0.400, and 0.844, and specificity was 0.859, 0.835, and 0.529, respectively. Imaging signs of bowel wall thickening, mesenteric edema, and fish tooth sign are valuable in predicting bowel wall ischemia, among which bowel wall thickening and mesenteric edema have relatively high specificity and fish tooth sign has a relatively high sensitivity. Furthermore, a fish tooth sign has the most favorable predictive value for bowel wall ischemia in acute intestinal obstruction, followed by bowel wall thickening and mesenteric edema.

## 1. Introduction

Intestinal obstruction, as one of the most common types of acute abdomen in the Emergency Department, accounting for about 15–20% of total cases of acute abdomen [1, 2]. In terms of location, intestinal obstruction may occur in small intestine and/or large intestine. Small bowel obstruction accounts for about 50–80% [3, 4], mostly resulting from adhesions [5, 6], and approximately 20–30% of patients require surgical intervention [7]. Large intestinal obstruction accounts for about 10–15% [8], which is mainly induced by tumors, and considering that it may form a closed loop [9], the majority of patients (about 75%) need surgical treatment [10, 11].

For the treatment of acute intestinal obstruction, international guidelines have always advocated conservation [12–14]. It has been reported that in the absence of clinical and/or radiological evidence of strangulation and intestinal ischemia, about 80% of intestinal obstruction cases can be successfully treated with conservative treatment [15]. However, intestinal obstruction has complex etiologies and various progressions, and if not treated promptly and effectively, it easily induces serious complications or even death [16]. Especially when blood supply disorders, the mortality rate can reach up to 10–35% [17–19]. Thus, identification of bowel wall ischemia at an early stage is crucial for making surgical decisions and also a great challenge for clinicians.

At present, a new imaging sign of bowel wall ischemia in intestinal obstruction has been discovered by our research team based on long-term clinical practice. In this study, the CT imaging signs that can predict bowel wall ischemia in intestinal obstruction patients were investigated via retrospective analysis on the 130 patients with intestinal obstruction who underwent surgery in our hospital, so as to establish the imaging prediction model of bowel wall ischemia in patients with intestinal obstruction.

## 2. Patients and Methods

### 2.1. Patients

The data of 302 patients diagnosed with acute intestinal obstruction in the General Surgery Department of the PLA Rocket Force Characteristic Medical Center from April 2016 to March 2022 were retrospectively analyzed. In total, 130 surgically treated patients met the inclusion criteria in this study, including 70 males and 60 females, with an average age aged (62.34 ± 16.11) years old, and they all had undergone CT examination before admission or surgery. The study was conducted by following the Declaration of Helsinki. This study was approved by the ethics committee of PLA Rocket Force Characteristic Medical Center. Signed written informed consents were obtained from the patients and/or guardians.

The inclusion criteria for acute bowel obstruction patients involved are as follows: (1) patients who underwent surgery in the Emergency Department, General Surgery Department, Gastroenterology Department, and Hepatobiliary Surgery Department for CT-proven intestinal obstruction, presenting with acute abdominal pain, abdominal distension, vomiting and/or cessation of defecation and exhaust, or those who received surgery for bowel obstruction, which was diagnosed by abdominal X-rays and reviewed by CT scan. (2) those with no bowel wall ischemia or necrosis detected during surgery. (3) those with bowel wall ischemia or necrosis, which was confirmed by surgical exploration or proven by histopathology.

Exclusion criteria were as follows: (1) patients who were clinically diagnosed with suspected intestinal obstruction and examined by X-rays or ultrasonography but not by CT scan, (2) those who were diagnosed with intestinal obstruction by CT scan but received no surgery, or (3) those with incomplete diagnosis and treatment process (e.g., patients without final diagnosis due to voluntary discharge during hospital stay).

### 2.2. CT Equipment and Scan Parameters

Prior to admission or surgery, all patients were examined by CT scan using a Discovery HD750 64-row spiral CT scanner (GE, USA) from bilateral diaphragmatic domes to symphysis pubes. Scan parameters were set as below: tube voltage: 120 kV, tube current: 220 mA, slice thickness: 2.5 mm, slice spacing: 7.5 mm, and reconstructed slice thickness and slice spacing: 2.5 mm. All images were stored in the PACS system workstation.

### 2.3. Image Analysis

All images were analyzed by 2 radiologists who had more than 10 years of experience on imaging analysis. Based on references about bowel ischemia, complex signs such as “closed loop”, “beak sign”, “whirl sign”, “cup mouth sign”, “strand sign”, and “target sign” were selected (Figures 1–6), signs of mesenteric edema, bowel wall thickening, bowel wall pneumatosis and ascites (Figures 7–10), and fish tooth sign (Figures 11 and 12) were analyzed.

### 2.4. Statistical Analysis

SAS software was used to assign values (yes = 1, no = 0) to all qualitative data of patients eligible in this study. Quantitative data were based on the original medical records and expressed as mean ± standard deviation ($\bar{\chi }$ ± *s*). Qualitative data were analyzed by *χ*^2^ test (Fisher's exact probability test was utilized in the case that all theoretical numbers were >1 and there was at least one theoretical number ≤5). *P* < 0.05was considered statistically significant. Variables with statistical significance were incorporated into multivariate logistic regression analysis. The relative risk and confidence interval (CI) of each variable were calculated, and the sensitivity, specificity, and positive likelihood ratio (LR+) and negative likelihood ratio (LR-) of the model in predicting intestinal wall ischemia in intestinal obstruction were evaluated.

## 3. Results

The clinical and imaging data of 302 patients with intestinal obstruction were retrospectively analyzed in this study. The patients were averagely aged (62.34 ± 16.11) years old and suffered from intestinal obstruction mostly resulting from adhesions (*n* = 134), followed by gastrointestinal tumors (*n* = 58), and the incidence rate of bowel wall ischemia was 14.90% (Table 1). A total of 172 patients received conservative treatment, while 130 patients underwent surgical treatment, of which 45 patients developed bowel wall ischemia. According to univariate analysis (*n* = 130), 5 factors with statistical significance were identified (Table 2), including bowel wall thickening, mesenteric edema, bowel wall pneumatosis, ascites, and fish tooth sign. Multivariate logistic regression analysis manifested that 3 factors entered into the prediction model (Table 3), including mesenteric edema, bowel wall thickening, and fish tooth sign. The model indicated that the predictive value of fish tooth sign for bowel wall ischemia in intestinal obstruction was the most notable, followed by bowel wall thickening and mesenteric edema. According to diagnostic evaluation on these 3 factors in the model, it was concluded that fish tooth sign had the highest sensitivity (0.844), followed by bowel wall thickening (0.400) and mesenteric edema (0.356) (Table 4).

## 4. Discussion

Acute intestinal obstruction is one of the most common forms of acute abdomen, characterized by acute onset and complex and varied conditions, and if not diagnosed and treated correctly or promptly, it will result in tremendous consequences [16]. As previously reported, approximately, 7–42% of intestinal obstruction patients are complicated with bowel wall ischemia [11]. The incidence rates of bowel wall ischemia in volvulus, intra-abdominal hernia, and closed-loop obstruction are 60%, 43%, and 43%, respectively, and that in simple adhesive intestinal obstruction is 21%, while no bowel wall ischemia is detected in malignancy-related intestinal obstruction patients [20]. In our study, the results demonstrated that intestinal obstruction complicated with bowel wall ischemia showed an incidence rate of 14.90%. Additionally, the incidence rates of bowel wall ischemia in intra-abdominal hernia, intussusception, incarcerated external abdominal hernia, and volvulus were about 92.30%, 50%, 35.71%, and 33.33%, respectively. The incidence rate of bowel wall ischemia in simple adhesive intestinal obstruction was about 12.59%, and that in malignancy-induced intestinal obstruction was about 6.56%, which may be attributed to late tumor stage, closed-loop bowel obstruction in some cases and mesenteric tumor thrombosis.

Currently, with a sensitivity and specificity of 94% and 96%, respectively, for the diagnosis of intestinal obstruction [21], multi-slice spiral CT(MSCT) imaging has been widely applied in clinical practice. Moreover, broad consensus has been reached on the value of CT imaging in assessing whether intestinal obstruction requires surgical intervention [22–28]. The comprehensive sensitivity and specificity are 87% and 73%, respectively, while two imaging signs are pivotal for determining whether it is necessary to perform surgical intervention, namely, local ischemia and complex signs [29]. Complex signs such as “closed loop”, “beak sign”, “whirl sign”, “cup mouth sign”, and “target sign” can be readily judged by experienced clinicians and radiologists, but it is difficult to evaluate the imaging of local bowel wall ischemia. Relevant data indicated that delayed surgery for intestinal obstruction with bowel wall ischemia markedly increases the mortality rate [29].

At present, bowel wall thickening, bowel wall pneumatosis, bowel wall density decline, mesenteric edema, ascites, and portal venous gas and inflation are recognized as CT imaging signs of local bowel wall ischemia [30]. In actual clinical practice, it is difficult to perform enhanced CT scan required for confirming partial imaging signs in real time, and even the illness of some patients may progress rapidly while waiting for enhanced CT examination. For this reason, obtaining local bowel wall ischemia signs through plain CT scan is particularly important. In this study, mesenteric edema, bowel wall thickening, bowel wall pneumatosis and ascites were screened out from imaging signs that can be obtained by plain CT scan of the abdomen. Additionally, a new imaging sign with potential relevance to bowel wall ischemia has been discovered by our research team based on long-term clinical practice, which is named “fish tooth sign”. Such sign can be obtained by a plain CT scan and was also included into the study. Compared with currently recognized signs of bowel wall ischemia, the sensitivity of “fish tooth sign” was the highest (84.44%), as reported in this study. Furthermore, the partial regression coefficient also suggested that “fish tooth sign” was the most significant predictor of bowel wall ischemia, which was greatly valuable for clinical guidance, while the findings were not identified in previous studies. In view of this, it is recommended that in the event that the “fish tooth sign” is present in patients definitely diagnosed with intestinal obstruction, regardless of the types, bowel wall ischemia should be highly suspected.

There were also some limitations in this study. First, it was uncovered that the “fish tooth sign” appeared in the obstructive segment or the proximal intestinal segment with relatively obvious pneumatosis and effusion, which might be related with early-stage inflammation in intestinal wall, microcirculation disorders and intestinal mucosal edema, and further research is needed for validation. Second, there might be a regional statistical bias in this single-center retrospective study, so prospective and multicenter studies are needed to verify the current research findings. Third, clinical data in this study might be biased, such as malignancy-induced intestinal obstruction, whose partial conclusion differed from that in foreign literature. Besides, owing to the limitation of the PACS system, there was a difficulty to acquire CT imaging data before 2016, which led to notable reductions in the total sample size and positive cases. In the following study, we will continue to conduct more case studies with multicenter cooperation in order to obtain more accurate data.

## 5. Conclusion

Currently, a consensus has not yet been reached on the indicators for determining surgery timing of intestinal obstruction, and most previous prediction models are extremely complex to be developed in many primary hospitals. However, the “fish tooth sign” proposed in this study has a higher sensitivity and is easy to be identified, which can greatly shorten the learning curve of clinicians and radiologists. Moreover, the prediction model is more convenient and valid, which is worthy of popularization, thus assisting clinicians to make surgical decisions.

## Figures and Tables

**Figure 1:** A 55 year-old male patient with adhesive intestinal obstruction. The CT image shows a closed loop. Bowel wall ischemia was seen during surgery.

**Figure 2:** A 61 year-old male patient with adhesive intestinal obstruction complicated with small intestinal volvulus. He had received surgery for rectal cancer 2 years ago. The CT image shows a beak sign in front of abdominal aorta. No bowel wall ischemia was identified during surgery.

**Figure 3:** A 78 year-old male patient with megacolon complicated with volvulus. The CT image shows a whirl sign. Bowel wall ischemia and mesenteric venous thrombosis were observed during surgery.

**Figure 4:** A 45 year-old male patient with intussusception caused by lipoma of the ileum. The CT image shows a cup mouth sign. No bowel wall ischemia was identified during surgery.

**Figure 5:** A 66 year-old male patient with paraduodenal hernia. The CT image shows a mesenteric strand sign. No bowel wall ischemia was identified during surgery.

**Figure 6:** An 88 year-old male patient with intussusception caused by stromal tumor of the small intestine. The CT image shows a target sign. Ischemic necrosis of the intestinal wall was seen during surgery.

**Figure 7:** A 22 year-old female patient suffered from uterine perforation caused by curettage surgery, and adhesive intestinal obstruction afterwards, which led to abdominal abscess and formation of internal ileal fistula. During surgery, partial bowel wall necrosis was seen at the fistula orifice.

**Figure 8:** A 75 year-old male patient with adhesive intestinal obstruction complicated with partial small intestinal volvulus. He had received “radical resection of rectal cancer”. The CT image shows bowel wall thickening proximal to the obstruction. During surgery, bowel wall ischemia was seen at the site of severe adhesion.

**Figure 9:** An 81 year-old female patient with internal hernia of the small intestine. The CT image shows incarcerated intestinal canal and wall pneumatosis. Ischemic necrosis of the incarcerated intestinal canal was seen during surgery.

**Figure 10:** A 48 year-old male patient with adhesive intestinal obstruction. He had received “radical resection of rectal cancer”. The CT image shows signs of ascites. Partial bowel wall ischemia of the small intestine proximal to the obstruction was seen during surgery.

**Figure 11:** A 55 year-old male patient with intra-abdominal hernia complicated with small intestinal volvulus. A fish tooth sign was seen in the intestinal canal proximal to the obstruction. Ischemic necrosis of the incarcerated intestinal canal was seen during surgery.

**Figure 12:** A 28 year-old female patient had received “appendectomy” and suffered from “intestinal obstruction” for several times after the operation. The CT image shows a fish tooth sign. Partial ileum and its mesenterium adhered to the abdominal wall of the incision, and no bowel wall ischemia was identified during surgery.

**Table 1:** Etiology and incidence rate of bowel wall ischemia in 302 patients with intestinal obstruction.

Etiology	*n*	Percentage (%)	Ischemia case	Incidence rate of ischemia
Adhesions	134	44.37	17	12.59
Intra-abdominal hernia	13	4.30	12	92.30
Volvulus	6	1.99	2	33.33
Intussusception	2	0.66	1	50.00
Incarcerated external abdominal hernia	14	4.64	5	35.71
Malignancy	58	19.21	4	6.90
Paralysis	13	4.30	0	0
Dynamics	32	10.30	0	0
Fecal stones	22	7.28	1	4.55
Mesenteric thrombosis	3	0.99	3	100
Others	5	1.66	0	0
Total	302	100	45	14.90

**Table 2:** Univariate analysis of CT signs of bowel wall ischemia in 130 patients undergoing intestinal obstruction surgery.

CT sign		Ischemia (*n* = 45)	Non-ischemia (*n* = 85)	*P*
Mesenteric edema	Yes	16	12	0.0047
	No	29	73	

Bowel wall thickening	Yes	18	14	0.0030
	No	27	71	

Bowel wall pneumatosis	Yes	5	2	0.0483^#^
	No	40	83	

Ascites	Yes	19	19	0.0178
	No	26	66	

Complex signs	Yes	18	39	0.5202
	No	27	46	

Fish tooth sign	Yes	38	40	<0.0001
	No	7	45	

^#^: Fisher's exact probability test.

**Table 3:** Multivariate regression analysis of CT signs and bowel wall ischemia in 130 patients with intestinal obstruction.

CT sign	Partial regression coefficient	OR	95% CI	*P*
Mesenteric edema	1.173	3.232	(1.112, 9.390)	0.031
Bowel wall thickening	1.129	3.093	(1.131, 8.459)	0.028
Fish tooth sign	2.164	8.707	(3.063, 24.752)	<0.001

#OR: odds ratio, CI: confidence interval.

**Table 4:** Diagnostic evaluation of CT signs of bowel wall ischemia.

CT sign	Se	Sp	LR+	LR-	YI
Mesenteric edema	0.356	0.859	2.525	0.750	0.215
Bowel wall thickening	0.400	0.835	2.424	0.719	0.235
Fish tooth sign	0.844	0.529	1.792	0.295	0.373

^#^Se: sensitivity, Sp: specificity, LR+: positive likelihood ratio, LR-: negative likelihood ratio, YI : Youden's index.

## Data Availability

The datasets used and analyzed during the current study are available from the corresponding author on reasonable request.
